The article "The majority of conversion total hip arthroplasties can be considered a primary replacement: a matched cohort study" was retracted in 2021. Reasons: plagiarism; duplicate publication.

# The majority of conversion total hip arthroplasties can be considered a primary replacement: a matched cohort study

**DOI:** 10.1186/s40001-020-00467-6

**Published:** 2020-12-11

**Authors:** Soufiane Aharram, Mounir Yahyaoui, Jawad Amghar, Abdelkarim Daoudi, Omar Agoumi

**Affiliations:** 1 Department of Trauma and Orthopaedics, University Mohammed Premier Oujda, Mohammed VI Oujda Morocco Hospital Center, Oujda University, BP 4806, 60049 Oujda, Morocco; 2 Faculty of Medicine and Pharmacy of Oujda, Department of Traumatology Orthopeadic Surgery, CHU Mohammed VI, Oujda University, BP 4806, 60049 Oujda, Morocco

**Keywords:** Proximal femur fracture, Total hip arthroplasty, Conversion, Primary, Revision, Matched cohort study

## Abstract

**Background and study aims:**

The success of conversion total hip arthroplasty (THA) among primary THA and revision THA remains unclear. We hypothesized that most conversion THA’s can be performed using primary implants and will have an uncomplicated post-operative course.

**Materials and methods:**

Thirty-six patients (23 females, mean age 68,0y) who underwent conversion THA for failed interventions for proximal femur fractures in the period 2008–2018 were matched sequentially against patients of the same sex and age who underwent primary THA or revision THA. Data were collected on implants used, major complications, and mortality. PROMs used included the Western Ontario and McMaster Osteoarthritis Index, Harris Hip Score, Visual Analogue Scale and the EQ-5D Health Questionnaire.

**Results:**

Seventy-two percent of patients who underwent conversion THA were treated with primary implants and never suffered from a major complication. PROMs were excellent for this group of patients. The distinction primary/conversion/revision THA could not explain differences in outcomes; however, the necessity of using revision implants and the development of major complications could.

**Conclusions:**

The majority of conversion total hip arthroplasties can be considered a primary replacement. Predicting outcomes for THA should focus on patient frailty and technical difficulties dealing with infection, stability and loss of bone stock and should discard the conversion versus revision terminology.

## Background

A primary total hip arthroplasty (pTHA) is most commonly performed for osteoarthritis (OA), usually has an uneventful post-operative course and is known for its excellent long-term results [1].

Nevertheless, failures do occur, for a variety of reasons, and are most often followed by a revision (r) THA. This is a technically more demanding procedure, revision implants are often necessary, and can range from changing a worn-out polyethylene liner in a not yet unstable hip to a two-stage revision for a difficult to treat infection with substantial bone loss. Results of rTHA’s are less favourable than those seen in pTHA’s due to the fact that complications are more common, survival of implants is shorter, and patients report lower on outcome measures (PROMs) [2–4].

A third group of hip replacements is made up by the conversion (c) THA’s. These are usually performed when an intervention for a proximal femur fracture has failed (Fig. 1) and is salvaged by THA [5–9]. Again, this a very diverse group as it can include patients undergoing placement of an additional cup in a hemi-arthroplasty (HA) that is causing painful erosion of the native acetabulum or patients with infected cephalomedullary nails with non-union, significant bone loss and an escaped abductor apparatus. Besides these technical difficulties, there frequently are concomitant medial issues as the typical patient requiring cTHA is of old age, has multiple health issues, and usually has been barely mobile in the period awaiting salvage surgery.

**Fig. 1:** Spectrum of failed hardware initially used to treat proximal femur fractures

Attempts have been made to determine the success of cTHA among pTHA and rTHA, as this has implications for patient consenting and institutional reimbursement [10–17]. It has been suggested that a cTHA should be considered an rTHA, but also that it is a distinct entity with outcomes in between pTHA and rTHA [13, 14, 16]. Interpreting these studies is difficult, as matched cohort analyses are rare, follow-up differs between groups, but most importantly because of the fact that very diverse groups of cTHA’s are compared to very diverse groups of rTHA’s [10–17]. This raises the question whether it is useful to predict outcomes based on this distinction in the first place [15, 16]. There is a subgroup of patients who undergo cTHA using primary implants, who will never develop any complications and whose satisfaction probably resemblances those of patient with pTHA’s [17].

We, therefore, performed a matched cohort study and formulated the following three hypotheses:

1. The distinction pTHA/cTHA/rTHA will not be able to explain differences in outcomes.
2. Necessity of revision implants and development of major complications will be able to explain differences in outcomes.
3. Most cTHA’s can be performed using primary implants and will have an uncomplicated post-operative course.

## Materials and methods

### Design

The theatre diaries of our dedicated hip unit were meticulously searched for patients who underwent cTHA for failed interventions for proximal femur fractures during the period from January 2008 to December 2018. They were matched sequentially against patients of the same sex and age who underwent pTHA or rTHA in the same year.

### Patients

Thirty-six patients (23 females, mean age 68,0 y (SD 14,0; 34–86), 24 left hips) who had undergone cTHA were identified (Table 1). There were 11 failed dynamic hip screws (DHS), 10 HA, 4 cephalomedullary nails, 9 cannulated screws, and 2 proximal femoral plates. All pTHAs were performed for OA. Indications for rTHA included a mix of infection, loosening, instability, polyethylene wear, leg length discrepancy and (peri)-prosthetic fracture. The primary conversion surgery cTHA is in the interval of 3 to 6 months. But the revision surgery rTHA was still after 2 years.

**Table 1:** Demographic data, mortality and PROMs of the three cohorts of hip replacements

	pTHA	cTHA	rTHA	F	p
*N*	36	36	36		
Sex (F, %)	23 (63.9%)	23 (63.9%)	24 (66.7%)		
Age fracture (mean)	NA	63,6 y (SD 14.8; 27–85)	NA		
Age p/cTHA (mean)	69.1 y (SD 12.4; 39–86)	68,0 y (SD 14.0; 34–86)	59,7 y (SD 14.6; 29–82)	4,177	0.8
Age rTHA (mean)	NA	NA	69,0 y (SD 12.8; 39–85)		
Side (L, %)	14 (38.9%)	24 (66,7%)	12 (33.3%)		
ASA (median)	2 (1–3)	2 (1–3)	2 (1–3)		
F/U (mean)	6.4 y (SD 4.3; 1,2–13,2)	6.4 y (SD 4.3; 1,2–13,2)	6,4 y (SD 4.3; 1,2–13,2)	0,000	1.00
VAS overall health (mean)	67.8 (SD 24.7; 20–100)	61.0 (SD 25.5; 20–100)	65,1 (SD 18.7; 30–99)	0,428	0.65
Major complications	4	4			
1 year mortality (%)	3 (8.3%)	1 (2.8%)	0 (0%)	1,828	0.17
Mortality at final F/U (%)	9 (25.0%)	7 (19.4%)	6 (16.7%)	0,391	0.68
WOMAC					
Pain (mean)	79.7 (SD 28.9; 20,0–100)	66.1 (SD 29.8; 0–100)	72,2 (SD 33.2; 0–100)	1,036	0.36
Stiffness (mean)	82.2 (SD 28.4; 12,5–100)	64.7 (SD 34.9; 0–100)	63,2 (SD 33.9; 0–100)	2,030	0.14
Difficulties (mean)	69.7 (SD 30.8; 7,4–100)	59.4 (SD 35.5; 0–100)	58,1 (SD 28.7; 0–97,1)	0,746	0.48
Total (mean)	72.7 (SD 29.0; 12,5–100)	61.8 (SD 32.5; 6,3–100)	61,6 (SD 29.1; 0–97,9)	0,850	0.43
EQ-5D					
Mobility (mean)	1.4 (SD 0.5; 1–2)	1.7 (SD 0.7; 1–3)	1,8 (SD 0.6; 1–3)	2,335	0.11
Self-care (mean)	1.5 (SD 0.6; 1–3)	1.5 (SD 0.7; 1–3)	1,8 (SD 0.5; 1–3)	1,513	0.23
Usual activities (mean)	1.7 (SD 0.7; 1–3)	1.7 (SD 0.8; 1–3)	1,9 (SD 0.5;s 1–3)	0,991	0.34
Pain (mean)	1.5 (SD 0.7; 1–3)	1.4 (SD 0.6; 1–3)	1,8 (SD 0.6; 1–3)	1,496	0.23
Anxiety (mean)	1.3 (SD 0.6; 1–3)	1.5 (SD 0.7; 1–3)	1,4 (SD 0.6; 1–3)	0,694	0.50
HHS					
Pain	75.8 (SD 32.3; 0–100)	67.6 (SD 31.7; 0–100)	68,2 (SD 33.4; 0–100)	0,396	0.68
Limp	75.1 (SD 30.9; 0–100)	56.5 (SD 41.4; 0–100)	52,5 (SD 38.4; 0–100)	1,976	0.15
Support	61.2 (SD 37.7; 0–100)	41.9 (SD 38.2; 0–100)	43,4 (SD 37.8; 0–100)	1,705	0.19
Walking distance	56.0 (SD 32.1; 0–100)	45.5 (SD 34.6; 0–100)	39,9 (SD 29.6; 0–100)	1,190	0.31
Stairs	55.3 (SD 34.9; 0–100)	45.7 (SD 32.6; 0–100)	37,5 (SD 30.0; 0–100)	1,378	0.26
Socks and shoes	63.2 (SD 40.3; 0–100)	67.4 (SD 41.6; 0–100)	63,9 (SD 37.6; 0–100)	0,068	0.93
Sitting	90.5 (SD 25.3; 0–100)	90.4 (SD 24.6; 0–100)	90,0 (SD 25.9; 0–100)	0,002	1.00
Public transport	68.4 (SD 68.4; 0–100)	60.9 (SD 49.9; 0–100)	33,3 (SD 48.5; 0–100)	2,657	0.08

Ontario and McMaster Osteoarthritis Index; EQ-5D = EuroQol 5-Dimensional Health Questionnaire. p/cTHA patient's age between primary and revision surgery

*F*  female, *L*  left, *THA * total hip arthroplasty, *ASA*  American Society of Anesthesiologists score, *F/U*  follow-up, *VAS*  Visual Analogue Scale, *WOMAC*  Western

### Outcome measures

Medical records and all available radiographs were reviewed and data were collected on implants used, major complications (DVT/PE, death during admission, dislocation, prosthetic joint infection, periprosthetic fracture, and loosening), mortality after 1 year and at final follow-up. Patients were contacted for an interview over the phone (experienced complications, Western Ontario and McMaster Osteoarthritis Index (WOMAC), Harris Hip Score (HHS), Visual Analogue Scale (VAS) and the EQ-5D Health Questionnaire). If after four attempts patients could not be reached, data were considered missing. Standardized sumscores for the WOMAC and domain index scores for the EQ-5D were calculated as per the respective instruction manuals. Total scores for the HHS could not be calculated as information on deformity and mobility was missing for the majority of patients. Therefore, percentages of domain scores were calculated, e.g. if a patient stated he had “marked pain, serious limitation of activities”, he scored 10/44 for the pain domain.

### Statistical analysis

Statistical evaluation was performed using IBM Statistical Package for the Social Sciences version 25. One-way ANOVA testing was used to compare means between the three cohorts for ratio and interval variables. If *p* ≤ 0.05 was encountered, subsequent independent sample *t *tests were used to see between which groups the statistically significant difference existed. Next, two new cohorts were created, i.e. patients who underwent surgery using primary implants and had an uncomplicated follow-up vs. patients who required revision implants and/or had an complicated follow-up, regardless of this being a pTHA, cTHA, or rTHA. PROMs were compared between these two groups using independent sample *t* tests.

## RESULTS

### Hypothesis 1: The distinction pTHA/cTHA/rTHA will not be able to explain differences in outcomes

Table 1 shows the baseline characteristics, mortality and PROMS of the three groups of patients. Cohorts were comparable for age, sex, year of operation, objective (ASA) and subjective (VAS) overall health scores, and duration of follow-up (Table 1). No statistically significant differences in mortality after 1 year (*p* = 0.17) or at final follow-up (*p* = 0.68) were found. Major complications were rare (Fig. 3d: 14 in total during 691 patients years of follow-up) and did not differ significantly between groups. PROMs were obtained for 19 of the pTHA patients (9 deceased, 8 missing), 23 of the cTHA patients (7 deceased, 6 missing), and 18 of the rTHA patients (6 deceased, 12 missing). Standardized WOMAC sumscores, EQ-5D domain index scores, and HHS percentage scores did not show statistically significant differences between the three cohorts (Table 1),

### Hypothesis 2: Necessity of revision implants and development of major complications will be able to explain differences in outcomes

Next patients were divided into 2 groups (Fig. 3e): patients who did not require revision implants and experienced no major complications during follow-up (“No”, *n* = 68) and patients who required revision implants and/or experienced major complications during follow-up (“Yes”, *n* = 40). Figure 2 illustrates the significant differences in all WOMAC sumscores, EQ-5D domain index scores, HHS percentage scores (except “sitting”) and VAS general health scores. Therefore, more difficult operations (i.e. the use of revision implants) and setbacks during follow-up (major complications) will influence PROMs.

**Fig. 2:** Multiple line charts of EQ-5D, WOMAC, HHS and VAS scores

### Hypothesis 3: Most cTHAs can be performed using primary implants and have an uncomplicated post-operative course

Figure 3 shows the amount of revision stems, revision cups and revision liners (constrained or dual mobility) used for the three groups of patients. For all pTHAs, primary implants had been used. Significant more revision stems (7 vs 19; *p* < 0.01) and revision cups (2 vs 7; *p* < 0.01) were deemed necessary for rTHA cases compared to cTHA cases. More revision liners were used in the rTHA group than in the cTHA group, but this did not reach statistical significance (*p* = 0.21). As can be seen in Fig. 3e, 26/36 (72%) patients who underwent cTHA were treated with primary implants and never suffered from a major complication. As already illustrated in Fig. 2, PROMs are high in this group of patients.

**Fig. 3:** Stacked bar charts of implants used and major complications

## Discussion

This study matched and compared a cohort of patients who underwent cTHA to patients who underwent pTHA and rTHA. Several conclusions can be made.

First, the distinction pTHA/cTHA/rTHA is not able to explain differences in outcomes. No significant differences in major complications, mortality or PROMs were found. We, therefore, propose to stop using this distinction when trying to predict complications, implant survival and costs. The type of primary implant, whether this is a nail, a plate, a HA or a THA, is not correlated to the outcome of redo surgery as this will yield very diverse groups and does not take into account more important predicting factors. In the present study, we found that the use of revision implants and the development of major complications could explain almost all differences seen in PROMs. The development and validation of a prediction model based on these and other parameters, e.g. patient frailty, the presence of pre-existent infection/instability, and significant bone loss, would be highly useful in daily clinical practice and for calculation of long-term costs for the society.

Second, we were able to perform most cTHAs using primary implants and most of them encountered no major complications during follow-up. We know that for this group of patients, costs are low and patient satisfaction is high, comparable to pTHA performed for OA. Other studies have reported similar mid-term results. Archibeck et al. reviewed 102 THA patients after failed internal fixation of a prior hip fractures [7]. Despite needing slightly more revision type femoral implants (32 vs 23% in the present study), they still had excellent outcomes with a mean HHS of 81.8 at last follow-up. Gjertsen JE et al. found that survival of the implants in the Norwegian Arthroplasty Registry 5 years after cTHA for failed internal fixation of femoral neck fractures was 96% [18]. Most recently, Morsi et al. reported on the clinical and radiological outcomes of converting aseptic failures of intertrochanteric fracture fixation using a dynamic hip screw (DHS) to a total hip arthroplasty (THA) in a single stage procedure. Standard straight, polished, collarless, cemented stems were used in all 107 cases. At an average follow-up of 7.4 years, they report 99% implant survivorship, a Harris Hip Score of 89.3 (range 71–95) and only a very small number of surgical complications [19].

We do realize that all our cTHA were performed within a high-volume arthroplasty unit with specialist hip surgeons and fellows. Contrary to proximal femur fractures that are ideally treated within 24 h and, therefore, often by the on-call team, it is our opinion that cTHAs should be performed by a dedicated hip surgeon, even if this means postponing the procedure.

This study has several limitations. Due to its retrospective nature confounding factors such as patient expectations were not investigated. McLawhorn et al. and Qun et al. found that patients who underwent cTHA required more transfusions, had longer operative times and length of hospital stays, and more often had non-home bound discharge [13, 15]. Due to the absence of these data, no cost analysis could be made. Although a period of 13 years was searched, still a relatively small cohort of cTHA patients was found, yet larger than reported in most studies [10–17]. Major complications could have been missed and not all patients were reached for questionnaire assessment.

In conclusion, predicting outcome and patient satisfaction based on the fact that the surgical procedure to be performed is a conversion rather than a revision is not useful. Nevertheless, most cTHAs can be performed using primary implants, and most patients report no major complications and high satisfaction.

## Data Availability

Not applicable.
